# MiR-451 Promotes Cell Proliferation and Metastasis in Pancreatic Cancer through Targeting CAB39

This article has been retracted.

**DOI:** 10.1155/2017/2381482

**Published:** 2017-01-19

**Authors:** Rende Guo, Jianhua Gu, Zhibin Zhang, Yi Wang, Chuan Gu

**Affiliations:** General Surgery Department, Tianjin First Central Hospital, Tianjin 300192, China

## Abstract

Emerging evidence shows that microRNAs (miRNAs) play important roles in the regulation of various biological and pathologic processes in human cancers and the aberrant expression of miRNAs contributes to the tumor development. In this study, our findings indicate that miR-451 is significantly overexpressed in pancreatic cancer tissues and cell lines and elevated expression of miR-451 contributes to promoted cell viability (in vitro and in vivo). Moreover, overexpression of miR-451 is closely linked to poor prognosis and lymphatic metastasis. Inhibition of miR-451 dramatically suppresses cell viability and invasion, promotes cell apoptosis, and induces cell cycle arrest. Furthermore, miR-451 directly targets CAB39 and negatively regulates its expression and inhibition of CAB39 contributes to the promoted cell viability and invasion. Our findings improve our understanding of the function of miR-451 in the identification and therapy of pancreatic cancer.

## 1. Introduction

Pancreatic carcinoma (PC) has one of the worst prognoses in malignant tumors with 39,590 deaths/year in the USA and 227,000 deaths/year worldwide [1, 2]. PC is typically asymptomatic at early stage and the disease becomes apparent at advanced stage with extensive local tumor invasion to surrounding tissues or distant organs which delay the treatment. For the moment, surgical resection seems to be the best option for the management; however the postoperative effect is not satisfactory with high recurrence and disappointing 5-year survival rate [3, 4]. Meanwhile, the treatment for PC based on chemotherapeutic drug, such as gemcitabine, contributes to the resistance to chemotherapy which leads to a poor prognosis of pancreatic cancer [5, 6]. Hence, it is urgent to identify a highly specific and sensitive tumor marker (especially for the early diagnosis of pancreatic cancer) for the therapeutic strategies [7, 8].

Emerging evidence indicates that the small (approximately 18–25 nucleotides) single stranded noncoding microRNAs (miRNAs) play important roles in the regulation of various biological and pathologic processes, including tumor growth and cell apoptosis [9–11]. It is well recognized that the alterations in the expression of multiple miRNAs are involved in the development of tumors via regulation of their target genes [12–16]. For example, microRNA expression profiling analysis identified more than 228 deregulation miRNAs in pancreatic cancer [17]. Studies conducted on miR-451 have provided evidence that miR-451 plays crucial role in diagnosis of human cancers including gastric cancer, colorectal cancer, and renal cell carcinoma [18–20]. However, the effect of miR-451 on cells is contradictory as Tsuchiya found that miR-451 contributed to the formation of basolateral polarity in epithelial cells while Bandres validated the fact that miR-451 was inhibited in colorectal cancer tissues. Particularly, recent studies suggest that miR-451 promotes glioma cell proliferation but reduces cell migration via targeting calcium-binding protein 39 (CAB39) through monophosphate-activated protein (AMPK) signaling pathway [21]. Moreover, some researchers suggested that miR-451 promoted mTORC1 activation by suppressing the expression of CAB39 and resulted in the suppression of LKB1 activity and its downstream substrate AMPK activation [21, 22]. In the present study, we investigated the potential roles of miR-451 in human pancreatic cancer cell lines and our findings suggested that miR-451 potentially targets CAB39 and elevated expression of miR-451 significantly promotes cell proliferation and invasion in pancreatic cancer cells.

## 2. Materials and Methods

### 2.1. Patients and Cells

Twenty pairs of pancreatic carcinoma patients and healthy controls (human pancreatic cancer tissues, PC; matched normal adjacent normal pancreatic tissues, NP) were enrolled from Tianjin First Central Hospital for the present study. All the patients had written informed consent and the experiment was approved by the committees of Tianjin First Central Hospital, Tianjin, China. The PC and NP tissues were immediately frozen in liquid nitrogen after resection. All cases had been confirmed by pathologic examination with two individual pathologists. We employed four human pancreatic cancer cells (PANC-1, AsPC-1, BxPC-3, and SW1990) and normal pancreatic cells (HPNE cell) to investigate the expression patterns of miR-451 and CAB39 in pancreatic carcinoma cells. The human pancreatic cancer cells were maintained in DMEM containing 10% FBS and antibiotics. The HPNE cells (immortalized cells) were cultured in well-defined cell culture medium as previously described [11]. All the cells were incubated at 37°C, with 5% CO_2_.

### 2.2. Plasmids and Transfection

The CAB39 mRNA and wild-type 3′-UTR of CAB39 mRNA were, respectively, amplified and cloned downstream of the pcDNA3.1 and pGL3-Basic Luciferase Reporter Vector (Promega, Madison, Wisconsin, USA) to construct pcDNA3/CAB39 and CAB39-3′-UTR-WT. We employed QuikChange Mutagenesis Kit (Stratagene, La Jolla, CA, USA) to generate the mutation of wild-type 3′-UTR of CAB39 mRNA to be subsequently cloned downstream of pGL3-Basic Luciferase Reporter Vector to develop CAB39-3′-UTR-Mut. The miR-451 mimics, anti-miR-451, si-CAB39, and their corresponding controls (miR-NC, anti-miR-NC, and si-NC) were purchased from Shanghai GenePharma (Shanghai, China). Transfection was performed with Lipofectamine 2000 (Invitrogen, Grand Island, NY, USA). Briefly, 10^6^ cells were seeded the day before and then cotransfected with miR-451 mimics (50 nM)/anti-miR-451 (100 nM)/si-CAB39 (100 nM) or corresponding control, respectively, which will be subjected to Western blot/qRT-PCR analysis at indicated time. The primer of miR-451 mimics is as follows: 5′-AAACCGUUACCAUUACUGAGUU-3′, 3′-CUCAGUAAUGGUAACGGUUUUU-5′; the primer of anti-miR-451 oligonucleotides is as follows: 5′-UUCUCCGAACGUGUCACGUTT-3′, 5′-ACGU GACACGUUCGGAGAATT-3′.

### 2.3. RNA Extraction, qRT-PCR, and Western Blot

The total RNA of tissues and cells were extracted using Trizol reagent (Invitrogen) and then reverse transcribed into cDNA with High Capacity cDNA Reverse Transcription Kit (Applied Biosystems, Foster City, California, USA) according to the manufacturer's instructions. The quantification of the miR-451 expression in tumor tissues and cells was carried out using SYBR Premix Ex Taq TM II kit (TaKaRa, Otsu, Shiga, Japan) on the Applied Biosystems 7500 Real-time PCR system (Life Technologies, USA). The fold changes were calculated and normalized to human U6 (internal controls) with 2^−ΔΔCT^ method. Western blotting was carried out according to the well-defined methods with anti-CAB39 (1 : 1000, Abcam, Cambridge, MA, USA) and anti-GAPDH (1 : 500, Abcam, Cambridge, MA, USA).

### 2.4. MTT Assays

The MTT assay was performed with Cell Proliferation Kit (KeyGen Biotech, Nanjing, China) according to the instructions. Briefly, the cells (PANC-1 and AsPC-1 cells) were transfected with miR-451 mimics/anti-miR-451 or corresponding controls (miR-NC and anti-miR-NC), respectively, and incubated for 48 h. After transfection, 10 *μ*l of 1x MTT was add to each well and subsequently incubated for another 4 h at 37°C. 150 *μ*l DMSO was add to each well after decantation of the supernatant. The optical density (OD) was determined at 570 nm using Multiskan MS (Labsystems, Finland). Each experiment was performed in quintuplicate.

### 2.5. Annexin V-FITC/PI Apoptosis Assay and Cell Cycle Distribution

We employed apoptosis assay and cell cycle analysis to investigate the effect of miR-451 on cell apoptosis and cell cycle distribution. The annexin V-FITC assay and cell cycle analysis were performed following the standard procedure of annexin V-FITC/PI apoptosis kit (KeyGen Biotech) and Cell Cycle Detection Kit (KeyGen Biotech) on flow cytometer (FACSAria™ III, USA) as described previously [23, 24].

### 2.6. Matrigel Invasion Assay

Cell suspension (200 *μ*l, 2-3 × 10^5^ cells/ml) was collected and add to upper chamber of Transwell filters (8 *μ*m; Millipore, Boston, Massachusetts, USA) after transfection with anti-miR-451 or anti-miR-NC. The Transwell filters were precoated with or without BD Matrigel (50 *μ*l, BD Biosciences). The medium of lower chambers contains 10% FBS working as chemoattractant. After incubation for 24 h, the cells on the lower surface (invaded cells) were collected, fixed (3.7% formaldehyde), stained (0.1% crystal violet), and counted under a microscope. We chose five visual fields randomly and imaged them. Each experiment was performed in triplicate.

### 2.7. Dual Luciferase Assay

3 × 10^4^ cells (PANC-1 cell) were cultured in triplicate in 24-well plates the day before transfection, followed by cotransfection of CAB39-3′-UTR-WT/CAB39-3′-UTR-Mut and miR-451/anti-miR-451 or miR-NC/anti-miR-NC at indicated concentration with Lipofectamine 2000. After incubation for 48 h, the cells were collected and detected by Luciferase Reporter Assay Kit (Promega, USA). The results were normalized to pRL-TK and pMIR-vector (internal control).

### 2.8. Pancreatic Cancer Xenograft Model

BALB/c nude mice (number 30; 4-5 weeks old) were purchased and randomly divided into two groups (Lv-miR-451 and Lv-NC) to test the function of miR-451 in vivo. Lentivirus was conducted by triple transfection of PANC-1 cells with 4 *µ*g of miR-451/miR-NC and 4 *µ*g of lentiviral vector using lipid transfection (Lipofectamine-2000/Plus Reagent, Invitrogen). Then the lentivirus was subcutaneously injected in the flank of the nude mice, respectively. The tumor volumes were monitored every three days with Vernier calipers. The tumor volume was calculated using a standard formula: length/2 × width^2^. When the tumor volume reached 500 mm^3^, the mice were sacrificed and the tumor was harvested and frozen in −80°C for the subsequent assays.

### 2.9. Statistical Analysis

The data was presented as means ± standard deviation (M ± SD). The statistical analyses were performed using SPSS 19.0 statistics software. Data comparisons used paired *t*-test and group comparisons used one-way analysis of variance (ANOVA). *P* ≤ 0.05 was considered as statistically significant differences.

## 3. Results

### 3.1. Overexpression of miR-451 Is Related to Poor Prognosis

We employed qRT-PCR to investigate the expression pattern of miR-451 in pancreatic cancer tissues and cells. The results suggested the expression of miR-451 was significantly promoted in the tumor tissues and cells relative to the normal adjacent samples and cells (*P* < 0.05, Figures 1(a) and 1(b)). We further conducted Kaplan-Meier curves based on miR-451 levels in patient specimens tending to explore the relationship between the expression of miR-451 and patients prognosis (Figure 1(c)). The median survival of high miR-451 group (13.21 ± 2.48 months) was obviously decreased compared with low miR-451 group (36.33 ± 5.56 months) (*P* = 0.003). Our findings indicated that patients with high levels of miR-451 may be subject to poor prognosis compared with low levels of miR-451. Moreover, we analyzed the association of metastasis and miR-451. The result showed that patients with an elevated miR-451 expression were more frequently associated with tumor invasion and metastasis (Figure 1(d)). These data revealed that miR-451 may be involved in the carcinogenesis of pancreatic carcinoma.

### 3.2. MiR-451 Promotes Cell Viability In Vitro and In Vivo

Since miR-451 is considered to be involved in the carcinogenesis of pancreatic carcinoma, we wanted to investigate the effect of miR-451 on cell viability. The expression of miR-451 in cells (PANC-1 and AsPC-1 cells) transfected with miR-451/anti-miR-451 or controls was confirmed by qRT-PCR. The expression of miR-451 in cells transfected with miR-451 mimics was upregulated almost 4-fold in PANC-1 cells and 6-fold in AsPC-1 cells, whereas anti-miR-451 group decreased almost 60% (*P* < 0.05, Figures 2(a) and 2(b)). The MTT data indicated that the viability of miR-451 group was significant increased whereas the viability of anti-miR-451 group was significant decreased (in PANC-1 cells) comparing to corresponding controls (*P* < 0.05, Figure 2(c)). The MTT result in AsPC-1 cells was consistent with PANC-1 cells (*P* < 0.05, Figure 2(d)). We next aim to explore the role of miR-451 in tumorigenesis in vivo. PNAC-1 cells transfected with LV-miR-451 or LV-NC were injected into the flank of nude mice. The tumor volume was calculated every three days which showed that the tumor volume of LV-miR-451 had grown faster than LV-NC group (Figure 2(e)). Three weeks later, we harvested the tumors and detected the miR-451 expression in the tumors. The qRT-PCR result suggested tumors of LV-miR-451 group exhibited an increased level of miR-451 compared with LV-NC group (*P* < 0.05, Figure 2(f)). All these findings support that miR-451 promotes cell viability in vitro and in vivo.

### 3.3. MiR-451 Suppresses Apoptosis and Blocks Cell Cycle Progression in PC Cells

We further employed annexin V-FITC/PI apoptosis assay and flow cytometry to identify the effect of miR-451 on the cell apoptosis and cell cycle in PC cells. As shown in Figure 3(a) inhibition of miR-451 (anti-miR-451) resulted in significant promoted cell apoptosis (11.33% in PANC-1 cells and 26.45% in AsPC-1 cells) compared with the control (anti-miR-NC) (*P* < 0.05). The cell cycle data indicated that the inhibition of miR-451 (anti-miR-451) induced G1/G2 arrest. As shown in Figure 3(b) the percentage of PANC-1 cells in G0/G1 phase increased from 23.55% to 48.74% while cells in S phase significantly decreased from 73.12% to 50.65% in the cells transfected with anti-miR-451. Consistent with this, the percentage of AsPC-1 cells (anti-miR-451 group) at G0/G1 phase increased from 19.23 to 48.26%, while the cells (anti-miR-451 group) in S phase decreased from 67.38% to 48.23%.

### 3.4. MiR-451 Promotes the Invasion of PC Cells

The effect of miR-451 on the PC cell invasive ability was tested by the Matrigel invasion assays. From Figure 4 we can see that the number of cells transfected with anti-miR-451 was obviously reduced (52% in PANC-1 cells and 54% in AsPC-1 cells; data not shown) compared with cells transfected with anti-miR-NC (*P* < 0.01). These results represented that the inhibition of miR-451 decreased the invasive ability of pancreatic tumor cell.

### 3.5. CAB39 Is the Direct Target of miR-451 in PANC-1 Cells

Bioinformatic analysis with TargetScan showed that CAB39 is a potential target of miR-451. We further performed Fluorescent Reporter Assay to predict the potential target of miR-451. The mutation of miR-451 binding site was shown Figure 5(a). The EGFP intensity of CAB39-3′-UTR-WT + miR-451 was blocked compared with CAB39-3′-UTR-Mut + miR-451 group while the EGFP intensity of CAB39-3′-UTR-WT + anti-miR-451 was increased compared with CAB39-3′-UTR-Mut + anti-miR-451 group (*P* < 0.01, Figure 5(b)). The group of cells transfected with CAB39-3′-UTR-WT/CAB39-3′-UTR-Mut + miR-NC/anti-miR-NC were controls. Meanwhile, we performed qRT-PCR and Western blot to investigate the association between miR-451 and CAB39. The mRNA and protein expression of CAB39 was obviously inhibited in miR-451 group compared with miR-NC group, and its expression was distinctly upregulated in anti-miR-451 group relative to anti-miR-NC group (*P* < 0.01, Figure 5(c), qRT-PCR; Figure 5(d), Western blot). Thus, our results demonstrated that miR-451 can directly target CAB39 via binding to its 3′UTR sequence.

### 3.6. The Effect of miR-451 Can Be Rescued by Overexpression of CAB39

To further identify whether miR-451 regulating cell invasion and proliferation was mediated by CAB39, we cotransfected pcDNA3/CAB39 or pcDNA3 and miR-451 mimics or miR-NC into PANC-1 cells. The results revealed that overexpression of miR-451 induced downregulation of CAB39 (pcDNA3 + miR-451 mimics group) can be rescued by transfection of pcDNA3/CAB39 (Figure 6(a)). Meanwhile, overexpression of CAB39 (pcDNA3/CAB39 + miR-NC) could inhibit the cell viability and invasion in PANC-1 cells compared with pcDNA3 + miR-NC group (*P* < 0.05, Figures 6(b) and 6(c)). Moreover, increased expression of miR-451 (pcDNA3 + miR-451 mimics group) induced cell viability and invasion can be rescued by overexpression of CAB39 (pcDNA3/CAB39 + miR-451 mimics group) compared with corresponding controls (pcDNA3 + miR-NC) (*P* < 0.05, Figures 6(b) and 6(c)). These results indicated that CAB39 was the functional target of miR-451 and miR-451 regulated pancreatic tumor cells viability and invasion via CAB39.

### 3.7. CAB39 Plays Suppressive Role in PC Tumorigenesis

Since the effect of miR-451 on PC cell viability and invasion was mediated by CAB39, we next aimed to study the role of CAB39 in PC tissues and cells. We performed qRT-PCR, MTT, and Matrigel Invasion Assay to investigate the role of CAB39 in PC tumorigenesis. The qRT-PCR data revealed that the expression of CAB39 was decreased in PC tissues compared with NP tissues (Figure 7(a)). Inhibition of CAB39 expression caused by transfection of si-CAB39 led to increased cell viability and invasion in PANC-1 cell (*P* < 0.05, Figures 7(b) and 7(c)). Thus, our data showed CAB39 may act as a tumor suppressing factor in PC development.

## 4. Discussion

Tumorigenesis is a complex process and various molecular mediators are reported to influences tumor behaviors, including proliferation, apoptosis, cell cycle, migration, invasion, and angiogenesis. Recently miRNAs, especially miRNAs relating to cell proliferation and metastasis, are considered to be novel biomarkers for tumor diagnosis and treatment. For example, the well-identified miR-21 is found to be involved in several tumors such as non-small-cell lung cancer, colorectal cancer, and breast cancer [25–27]. MiR-21 is always upregulated in tumors and closely linked to poor prognosis. Overexpression of miR-21 contributes to cell migration and induces resistance to chemotherapy via regulating its target gene [28–30]. The potential roles of miRNAs in the treatment of pancreatic carcinoma have also been investigated. MiR-155 is reported to be used as an early diagnostic biomarker in pancreatic ductal adenocarcinoma and overexpression of miR-155 results in an inhibition of TP53INP1 which is involved in PC tumor development [31].

MiR-451 is found to play vital role in diagnosis of human cancer; however the regulation behavior is always complicated. MiR-451 is identified to control the regulation of glioma cell proliferation and migration through LKB1- AMPK signaling in glioblastoma [20, 32]. The microarray analysis reveals that miR-451 is increased in plasma of gastric cancer patients and decreased in postoperative samples which can be used as blood-based biomarkers for gastric cancer screening [33]. However, there are findings different from above. The ultradeep sequencing profiles with high-throughput SOLiD identified a downregulated miR-451 in human gastric cardia [20]. The expression level of miR-451 is also repressed in the serum of renal cell carcinoma patients with the sensitivity of 81%, specificity of 83%, and AUC of 0.86 [34]. Moreover, miR-451 exhibits a tumor-suppressive function in human glioma cells via inhibition of cell invasion and the expression of related protein [35]. All these data show that miR-451 is involved in various tumor developments through different regulation behavior and the exact role of miR-451 in tumorigenesis remains to be studied.

In the present study, we found that miR-451 was overexpressed in the pancreatic cancer tissues and four pancreatic cancer cell lines (PANC-1, AsPC-1, BxPC-3, and SW1990) compared to the normal adjacent tissues and normal cell line (HPNE cell). The expression of miR-451 was intimately linked with metastasis and poor prognosis in PC patients. Overexpression of miR-451 resulted in a promoted cell viability and invasion, whereas decreased expression of miR-451 led to inhibited cell viability and invasion, promoted cell apoptosis, and induced cell cycle arrest. Moreover, elevated miR-451 contributed to the promotion of tumor growth in nude mice. Studies have provided evidence that miR-451 is involved in the progression of tumors through promotion of mTORC1 activation and miR-451 suppresses the expression of calcium-binding protein 39 (CAB39) in human glioma [22, 36]. In this study, our data confirmed that miR-451 can directly target the 3′UTR of CAB39 and regulate the expression of CAB39 conversely. Inhibition of CAB39 contributed to the promoted cell viability and invasion. However, whether miR-451 is involved in pancreatic cancer through CAB39-mTORC1 activation needs our further investigation.

In conclusion, our results showed that miR-451 promoted cell viability and invasion through downregulation of CAB39. Further investigation of the exact mechanism under miR-451/CAB39 axis in pancreatic cancer would shed new light on the pathogenesis of pancreatic cancer and provide us new treatment approach for pancreatic cancer.

## Figures and Tables

**Figure 1:** The expression level of miR-451 in pancreatic cancer tissues and cell lines. (a) The expression level of miR-451 in pancreatic cancer tissues and normal pancreatic tissues as determined by real-time PCR. (b) The expression level of miR-451 in pancreatic cancer cell lines PANC-1, AsPC-1, BxPC-3, and SW1990 by real-time PCR. (c) The overall survival (OS) rates were estimated by the Kaplan-Meier method. According to the level of miR-451 expression, Kaplan-Meier OS curves of pancreatic cancer patients showed that a high expression of miR-451 was significantly correlated with poor prognosis. (d) miR-451 high expression correlated with lymphatic metastasis. ^*∗*^*P* < 0.05.

**Figure 2:** The effect of miR-451 on cell viability in vitro and in vivo. (a) The expression of miR451 in PANC-1 and AsPC-1 cells transfected with miR-451 or miR-NC. (b) The expression of miR451 in PANC-1 and AsPC-1 cells transfected with anti-miR-451 or anti-miR-NC. The cell viability in PANC-1 (c) and AsPC-1 cells (d) transfected with miR-451, anti-miR-451, miR-NC, and anti-miR-NC. (e) The tumor volume in xenograft tissues in vivo. (f) The expression level of miR-451 in xenograft tissues detected by real-time PCR; ^*∗*^*P* < 0.05.

**Figure 3:** Suppressing miR-451 accelerates cell apoptosis and induces the cell cycle arrest. (a) Suppressing the expression of miR-451 accelerates cell apoptosis rate in PANC-1 and AsPC-1 cells. (b) The effect of inhibition of miR-451 expression on the distribution of cell cycle in PANC-1 and AsPC-1 cells determined by flow cytometry analysis; ^*∗*^*P* < 0.05.

**Figure 4:** Inhibition of miR-451 suppresses invasion in PANC-1 and AsPC-1 cells. Representative fields of the invasive cells (PANC-1 and AsPC-1 cells) on the membrane are presented (200x magnifications); ^*∗∗*^*P* < 0.01.

**Figure 5:** CAB39 is the potential target gene of miR-451. (a) The target sites for miR-451 in the 3′UTR of CAB39 and the mutant target sites. (b) The EGFP Fluorescence Reporter result of PANC-1 cells cotransfected with CAB39-3′UTR/CAB-3′UTR-mutor miR-451/anti-miR-451 or miR-NC/anti-miR-NC. The expression levels of CAB39 mRNA in PANC-1 cells transfected with miR-451/anti-miR-451 or miR-NC/anti-miR-NC level determined by qRT-PCR (c) and Western blot (d); ^*∗∗*^*P* < 0.01 and ^*∗∗∗*^*P* < 0.001.

**Figure 6:** miR-451 rescue experiments in PANC-1 cells. (a) The expression of CAB39 in PANC-1 cells cotransfected with pcDNA3/CAB39/pcDNA3 and miR-451/miR-NC. (b) The cell viability of PANC-1 cells cotransfected with pcDNA3/CAB39/pcDNA3 and miR-451/miR-NC. (c) The invasive cell number of PANC-1 cells cotransfected with pcDNA3/CAB39/pcDNA3 and miR-451/miR-NC; ^*∗*^*P* < 0.05.

**Figure 7:** The expression level of CAB39 in pancreatic cancer tissues. (a) The expression level of CAB39 in pancreatic cancer tissues and normal pancreatic tissues determined by real-time PCR. (b) The effect of knockdown CAB39 by transfection of si-CAB39 on cell viability in PANC-1 and AsPC-1 cells. (c) The effect of knockdown CAB39 by transfection of si-CAB39 on cell invasion in PANC-1 and AsPC-1 cells; ^*∗*^*P* < 0.05.
